# Impact of low-carbon economic policies on the corporate environmental responsibility model in China

**DOI:** 10.1371/journal.pone.0314589

**Published:** 2025-01-17

**Authors:** Hongya Liu, Haslindar lbrahim, Meijing Song

**Affiliations:** 1 School of Management, University Sains Malaysia, Penang, Malaysia; 2 Hua Xin College of Hebei Geo University, Shijiazhuang, China; 3 School of Finance and Economics, Hainan Vocational University of Science and Technology, Haikou, China; Xi’an Jiaotong University City College, CHINA

## Abstract

This study investigates the impact of low-carbon economic policies on Corporate Environmental Responsibility (CER) in Chinese A-share listed companies, with a particular focus on the role of financing constraints as a mediating factor. Despite a decrease in environmental pollution incidents in 2022, the economic and social impacts of such incidents remain significant, highlighting the need for stronger environmental governance. Building upon previous research, this study utilizes data from the Shanghai and Shenzhen stock exchanges (2010–2020) and employs a Difference-in-Differences (DID) model to assess the effects of low-carbon economic policies introduced in 2016 on CER. The findings reveal that these policies positively influence CER and that financial constraints act as a mediator. The study finds how low-carbon policies indirectly promote environmental commitments by alleviating financial barriers. The research provides valuable insights for policy formulation, advocating for intensified reforms on the financial supply side to foster a sustainable economic framework. Additionally, it underscores the importance of implementing robust low-carbon policies to elevate corporate environmental responsibility. However, the study also notes limitations related to data scope and potential external factors influencing the results. These findings contribute to the broader discourse on sustainable development, offering a blueprint for harmonizing economic growth with environmental preservation and informing future research in this area.

## Introduction

Environmental pollution incidents have had a profound impact on both people’s daily lives and their ability to engage in normal production activities [1]. From 2005 to 2020, China made significant progress in reducing its carbon emissions per unit of GDP, a key indicator of its low-carbon transition. The Chinese government has shifted its focus to renewable energy resources, thereby reducing carbon emissions [2]. The initiatives include stricter environmental regulations, investments in renewable energy, and improvements in energy efficiency. By 2020, China’s carbon intensity had decreased by over 48% compared to 2005 levels, demonstrating substantial strides towards meeting its climate commitments and transitioning towards a more sustainable economic model [3]. Strict lockdowns and a decline in economic activity during the COVID-19 outbreak also caused China to temporarily reduce its carbon emissions. Satellite data shows a significant decrease in nitrogen dioxide levels, primarily due to reduced industrial output and transportation. This decrease in emissions was only temporary, though, since economic activity soon resumed. The pandemic emphasized that while legislative initiatives and behavioral adjustments may be used to benefit the environment temporarily, long-term emission reductions necessitate long-term, systemic changes [4]. Following COVID-19, China had a rebound in carbon emissions as economic activity picked back up. Attempts to boost the economy resulted in more energy and industrial production, undoing some of the environmental improvements made during the pandemic. The experience does, however, reveal the possibility of using sustainable recovery measures to reduce future emissions and foster robust economic growth that is in line with environmental objectives [5]. Examples of these tactics include investing in green technologies and enacting laws supporting low-carbon development. China has committed to reducing carbon intensity by 60–65% from 2005 levels by 2030, demonstrating a strong effort towards low carbon emissions and supporting the sustainable development goals [6].

According to investigations by the Ministry of Environmental Protection, although the number of environmental pollution incidents in 2022 decreased by 20.56% compared to 2021, 190 incidents still occurred, with 3 classified as highly severe and 5 as relatively severe. Authorities recorded 182 incidents with relatively lesser impact. These sudden environmental events have caused significant economic losses and casualties, significantly disrupting people’s lives and adversely affecting their quality of life [7].

According to the latest statistics from the China Securities Association, as shown in Fig 1, a total of 1,178 listed companies disclosed their environmental and social responsibility information in 2021. Among the 1,415 companies with valid samples, accounts for 83.25%, showing an increase of 17.67% compared to the disclosure rate (70.75%) in 2020. The remaining 237 companies did not disclose carbon information, accounting for 16.75%. While the disclosure rate of carbon information has increased, there is still significant room for improvement. The overall average score for greenhouse gas environmental performance in these 1,415 listed companies in 2021 was 27.6%. Among them, 569 companies scored above the average, accounting for 40.21% of all companies, representing a 55.06% increase compared to 2020 which was 17.80% [8]. By actively disclosing more accurate and comprehensive environmental and social responsibility information, listed companies can help investors accurately assess the company’s future sustainability and fulfill their environmental responsibilities.

**Fig 1:** Number of enterprises and the average score of carbon information disclosure rate in Shanghai and Shenzhen.

In 2016, the Chinese government initiated a strategic program of Comprehensively Promoting Energy Conservation and Emission Reduction, which put forward a series of policies and measures aimed at achieving sustainable economic growth by managing carbon emissions, promoting green and low-carbon development, and promoting efficient energy use. The core objective of the policy is to reduce carbon emissions and mitigate the impact of climate change. By enhancing carbon emissions management, promoting green and low-carbon technologies and products, and advancing clean and renewable energy development, it is possible to effectively reduce atmospheric pollution and environmental impacts. [9] found that green mergers and acquisitions of heavily polluting enterprises can effectively improve their risk-bearing ability; [10] combined green finance, and social responsibility theory with green growth theory, and studied the problem of financial institutions assuming environmental responsibility. [11] proposed that when managers make and disclose investments while emphasizing their social benefits rather than just company costs, investors respond positively. In recent years, scholars, both domestically and internationally, have made significant contributions to the research on corporate environmental responsibility (CER). They have summarized the concept and dimensions of CER. [12] explored the influences of factors such as environmental regulations, corporate environmental performance [13], environmental regulation and CSR green innovation [14] and CSR on corporate environmental performance using environmental strategy and green innovation as mediators [15], economic activities, climate change, and carbon risks [16] low-carbon city policy and environmental performance [17]. Researchers have pointed out that CER and environmental awareness play a key role in improving corporate reputation [18, 19], helping companies gain competitive advantages [20], and enhancing financial performance [21].

Although the above-mentioned studies have provided analyses of CER from multiple perspectives, there is still a lack of research on the relationship between environment-friendly policies and CER. Most of the existing studies focused on how institutional pressures impact corporate social responsibility, demonstrating that institutional forces positively affect CSR [22, 23]. Due to its exponential industrial growth, China is facing the issue of a heavy emission rate. In this regard, the Chinese future commitments to achieve carbon neutrality by 2060, create a critical need for the study to understand how the low-carbon emission policies can affect corporate environmental responsibility. Analyzing the impact of such sustainable policies on businesses or the environment provides richer insights into how Chinese firms are responsibly working to meet sustainable development or climate goals. The study contributes to the understanding of low–carbon policies and sustainable efforts. Additionally, some studies highlighted the mechanism affecting CER through subjective measures like questionnaires [24], but the phenomenon is still under-researched using solid objective measures. Such studies have limited generalizability due to potential biases, subjectivity and sample size adequacy. This study further introduces an indirect relationship through financing constraints. The link between low-carbon policies and CER has been discussed in previous studies [25], but the Chinese context and the mediation of financial constraints is a novel way to better shape the effectiveness of the policies. Financial constraint is a barrier to sustainability drives and it can limit firms’ ability to meet environmental responsibility. The mediation of financial constraints identifies the attention to the financial aspects of sustainability which needs not to be overlooked in policy matters. The study offers both academic and practical implications for researchers and policymakers, offering them a valuable understanding of how low-carbon policies can better shape corporate environmental responsibility amidst the global drives of sustainable development. The study extends academic literature on low-carbon economic policies, corporate environmental responsibility, institutional economics, and financial hurdles in innovation and innovation policy, and offers practical insights for environmentalists, policymakers and business leaders.

## Theoretical background

### Institutional theory and Porter’s hypothesis

The Nobel laureate, Douglass C. North clarified that institutions are like "rules of the game" in any society, covering both formal laws and rules and informal norms like customs, rituals and traditions. This work set the institutions theory. The institutions represent structures that provide the basis for human interaction and economic performance which help reduce uncertainty, guide behavior, and offer a framework for individuals and organizations to operate [26]. The institutional theory referring to the formal rules, informal norms, and practices [27] can better prove a structured formwork to explain how the external low-carbon economic policies influence corporate environmental behavior and performance.

The New Institutional Economics (NIE), a theory from economics, originated from Keith’s 1937 article "The Nature of the Firm" which extends the theory of traditional economics by integrating institutions (formal and informal) into the analysis. The new field was developed to enrich traditional economics by institutions that were often overlooked in previous economic outcomes [28]. It mainly focuses on the relationship between institutions, individuals, and economic activities, and introduces concepts such as property rights and transaction costs. This approach studies the composition and operation of institutions from innovation, technology and economic perspective [29]. The NIE framework suggests that the formation and implementation of low-carbon economic policies have different costs (like environmentally friendly technology, regulations etc.) which consequently shapes corporate environmental behavior [30]. The low-carbon economic policies represent institutions that set the behavioral norms and requirements for businesses and environmental protection. As a form of institutional pressure, low-carbon economic policies directly impact the behavior and decision-making of businesses through measures such as regulations, taxes, and incentives. To comply with policy requirements, businesses need to develop environmental strategies, invest in eco-friendly facilities and technologies, and reduce carbon emissions [31]. This institutional pressure provides intrinsic motivation to businesses thereby changing their stock trading behavior [32] and shifting towards more environmentally friendly and sustainable business models.

Another relevant hypothesis is the Porter Hypothesis, proposed by Michael Porter, which explains that designing environmental regulations can lead to innovation and better environmental performance and in turn help gain a competitive advantage [33, 34]. Contrary to the conventional viewpoint that it will increase the costs, Porter argued the regulations drive innovation, making companies more competitive and efficient in the long run [35]. Neoclassical economists believed that implementing environmental protection policies would increase production costs and reduce business competitiveness. This viewpoint argues that environmental protection and economic development cannot occur simultaneously [36]. However, scholars such as Porter and Linde [34] proposed a theory to counter the neoclassical perspective on environmental protection policies. They argue that appropriate environmental regulations can promote CER. There are two key premises of the Porter Hypothesis: First is that Environmental Regulations motivate Innovation rather than a hindrance thus shifting from a static to a dynamic model. Secondly, the Innovation benefits can offset compliance costs which will improve the firms’ competitive advantages.

This study further highlights the Porter hypothesis and institutional theory in the new context of Chinese firms. The study presents how Chinese firms comply with regulations while dealing with financial constraints. The innovation-driven viewpoint of the Porter Hypothesis in conjunction with the institutional perspective provides a unique way to understand how low-carbon economic policies drive corporate environmental behavior. The study explores how access to financial resources influences firms’ ability to observe environmental regulations. This perspective identifies that while low-carbon economic policies encourage innovation, firms with financial constraints may struggle to invest in environment-friendly technologies or processes.

### Hypotheses development

#### Low carbon economy and CER

The term “low-carbon economy” implies reducing carbon emissions and controlling environmental pollution while pursuing improved economic benefits [37]. Low carbon economy and corporate environmental responsibility (CER) are closely connected because firms’ role in mitigating carbon emissions and promoting sustainable practices are imperative. Businesses can accomplish carbon reduction targets, incorporate sustainability into their operational models, and comply with environmental regulations [38]. CER heightens firms’ reputations, drives innovation, and gives a competitive advantage by meeting stakeholder demands for environmental and financial accountability. Wan, Zhang [25] stated that companies need to manage their environmental performance that increase their CER and goodwill.

As a response to global climate change and environmental challenges, the concept of a low-carbon economy first emerged in 2003 in the UK government’s energy report titled “Our Energy Future—Creating a Low Carbon Economy.” In 2006, the Stern Review explicitly suggested that investing 1% of the Gross Domestic Product (GDP) per year could avoid future GDP losses of 5% to 20%, advocating for countries to transition to a low-carbon economy [39]. In 2007, the Chinese government released the “National Climate Change Program,” which set targets and policy measures to reduce carbon emissions, including energy conservation, optimizing energy structure, and promoting low-carbon technology adoption [40].

To develop a low-carbon economy, various approaches can be taken, such as controlling carbon emissions at the source through the development of clean energy, reducing pollution through technological innovation, and promoting the optimization and upgrading of industries through the development of low-carbon industries. Technological innovation, institutional innovation, innovative development models, and changes in people’s lifestyles can be formed as a result of a low-carbon economy [41]. Rather than the passive approach of polluting first and controlling later, the viable strategies now proactively take measures to control pollution during the development process, aligning with China’s strategic goal of sustainable development [42].

According to institutional theory, low-carbon economic policies serve as environmental regulations imposed by the government, imposing certain constraints and incentives on businesses. These policies possess varying degrees of coerciveness and normativity. Under government guidance, companies can improve their environmental performance by complying with relevant regulations and mandatory constraints. As mentioned by [43], environmental regulations and institutions can encourage companies to invest in corresponding environmental technologies to enhance their environmental performance. Scholars such as [44, 45] have emphasized the important role of the government in improving corporate environmental behavior. From the perspective of institutional constraints, low-carbon economic policies can passively induce businesses to fulfill their social responsibilities towards the environment.

In 2016, China initiated a nationwide pilot carbon market to reduce carbon dioxide emissions and incentivize the adoption of low-carbon technologies and clean energy through carbon emission trading mechanisms. Seven provinces and municipalities, namely Beijing, Shanghai, Chongqing, Tianjin, Guangdong, Hebei, and Hainan, implemented the pilot carbon market [46]. These regions pioneered the carbon market pilot by establishing carbon emission trading markets, encouraging companies to reduce carbon emissions, and utilizing carbon trading mechanisms to assess performance and implement punitive measures to promote low-carbon economic development.

Fulfilling CER can enhance corporate reputation [47], and companies can gain social capital through a positive reputation by signaling their responsible behavior [48]. According to stakeholder theory, the government is one of the stakeholders of the enterprise’s sustainable drives. When the government proposes to strengthen environmental protection in pilot areas through low-carbon economic policies, companies can cater to the government’s preferences by fulfilling their environmental and social responsibilities. This can enhance their legitimacy, establish a good reputation, and send signals to the government to gain support and resources [49]. On the other hand, if any government establishes a commitment to get environmental protection by initiating low-carbon economic policies, but firms fail to meet their environmental responsibilities, the stakeholders can notice such non-cooperative behavior [50]. In such cases, the stakeholders may "punish" the companies by reducing or withdrawing their support. In such cases, the implementation of low-carbon economic policies can also increase companies’ level of environmental social responsibility. This conclusion is not limited to the government as a stakeholder; it also applies when other stakeholders show concerns for environmental protection.

Once the government establishes low-carbon economic policies, external sources, such as the media, may pay more attention to the environmental quality in the policy-implementation regions. [51] projected that media attention can create a legitimacy crisis for firms and the attention may prove a source of their legitimacy that will grab the support of the government and stakeholders. [52] explored the relationship between media attention and corporate environmental investment and found that media attention can increase companies’ environmental investments. Therefore, the increased external attention received from the implementation of low-carbon economic policies may encourage companies to pay more attention to environmental protection issues and fulfill their social responsibility towards the environment. Based on these considerations, we propose the following hypothesis:

**Hypothesis 1**: *The implementation of low-carbon economic policies is positively related to the fulfillment of corporate environmental responsibility*.

#### Role of financing constraints as a mediator

Companies’ financial situation can considerably influence their response to environmental regulations and responsibilities. To clarify the theoretical basis as to why low-carbon economic policy influences environmental responsibility, Porter and Linde [34] viewed that appropriate environmental regulations can stimulate firms’ innovation activities, thereby impacting their competitiveness. Subsequent research strengthened the understanding of the Porter Hypothesis by finding that firms can affect their productivity [53], and improve their operational performance [54] by increasing innovation activities.

Some studies indicate that financing constraints can mediate the relationship between firms and environmental responsibility because financial limitations restrict firms’ ability to respond to or comply with environmental regulations [55]. Different mechanisms can mediate the effects of financing constraints on firms’ environmental responsibility. One involves the issue of cash flow. By limiting firms’ cash flow, financing constraints affect their financings and investments related to environmental protection [56]. Another mechanism relates to firms’ reputation and sustainable development goals. Financing constraints affect firms’ reputation and market position, which, in turn, affect their efforts and performance in environmental responsibility. Some research suggests that other factors can influence firms’ environmental responsibility under financing constraints. For example, factors like firms’ management capabilities, resource availability, and market competitiveness, which are related to environmental responsibility, may mediate the relationship under financing constraints, thus influencing firms’ environmental responsibility [55, 57, 58]. At the same time, firms’ environmental responsibility may also have a feedback effect on financing constraints. Some studies suggest that firms actively fulfilling environmental responsibility are more likely to obtain better financing conditions and opportunities for equity financing, thereby alleviating financing constraints. This feedback effect may further influence firms’ environmental responsibility behavior. Based on the arguments, we propose Hypothesis 2.

**Hypothesis 2**: *Financing constraints mediate the relationship between low-carbon economic policy and firms’ environmental responsibility*.

### Conceptual model

This study reviews the relevant literature on low-carbon economic policy and CER, identifying two main theoretical frameworks related to the research question: stakeholder theory and institutional theory. The theoretical background is based on the notion of clarifying the relationship between low-carbon economic policy and the fulfillment of environmental responsibility, as well as identifying the mediating mechanisms through which low-carbon economic policy influences CER. The study predicts a positive correlation between low-carbon economic policy and the level of CER, suggesting that companies can effectively enhance their fulfillment of environmental responsibility by implementing low-carbon economic policies. The study also posits that financing constraints mediate the relationship between low-carbon economic policy and the fulfillment of CER. By increasing financing constraints, the implementation of low-carbon economic policy can enhance companies’ fulfillment of environmental responsibility. Fig 2 depicts the conceptual model for this study.

**Fig 2:** Conceptual model.

## Research design

This study employs quantitative analysis to examine the relationship between low-carbon economic policy and corporate environmental responsibility (CER). Utilizing statistical methods, the researchers analyze large datasets, identifying trends, patterns, or correlations among different variables. For instance, researchers use regression analysis to assess the impact of specific policy interventions on corporate environmental performance indicators. Researchers employ econometric techniques to establish causality and estimate the effect of low-carbon policies on CER. These methods aim to control for confounding factors and address endogeneity issues [52]. Researchers often use panel data or instrumental variable approaches to isolate the effects of policy interventions, independent of other factors that may influence environmental responsibility.

### Sample selection and source of data

As China’s economy and society continue to develop, the scale of listed companies in the Shanghai and Shenzhen stock exchanges has been expanding, and their quality has improved gradually. They have strengthened their role in the operation of the national economy. Listed companies have become the main force in China’s economy, and their environmental responsibility is representative.

The CER Index quantitatively measures the performance of CER [59, 60]. Due to the different industries and business operations of companies, the indicators used to quantify environmental responsibility may vary among different companies. From the existing literature [61], there are generally two methods for quantifying the performance of CER. The first method is for researchers to establish their index system for environmental responsibility and collect data based on this system to calculate the companies’ environmental responsibility index. The second method is to directly use the environmental responsibility index published by other organizations for research purposes. Before 2009, few institutions in China calculated the environmental responsibility index of Chinese companies. However, after 2009, with the popularity of corporate social responsibility research, some institutions started to calculate the CER index [62]. Among them, the most representative ones are the CSR Blue Book published by the Chinese Academy of Social Sciences and the listed company environmental responsibility index published by Hexun.com, which includes the calculation of the environmental responsibility index for companies listed on the Shanghai and Shenzhen stock exchanges [63].

The sample for this study consists of companies listed on the Shanghai and Shenzhen stock exchanges from 2010 to 2020. Financial indicators and data on the executive teams are sourced from the CSMAR database and Hexun’s corporate social responsibility reports. The environmental responsibility scores of companies are obtained from Hexun.com. Researchers merge the two sets of data based on company names, excluding missing observations, ST, *ST, and PT-listed companies, as well as those with abnormal calculations of equity capital. Finally, a panel dataset with 3,799 observations is selected. The study sources data on environmental regulation intensity from the “China Statistical Yearbook” and obtains data on social supervision from the City Pollution Source Environmental Disclosure Index.

### Variables selection

#### Dependent variable

Researchers can use two types of data when conducting empirical research on CER. Firstly, scholars may use content analysis to quantitatively assess the environmental responsibility of companies. Scholars develop their evaluation index system based on authoritative social responsibility standards such as ISO 26000 and ESG (Environmental, Social, and Governance) guidelines [63]. They then use surveys or information disclosed by companies to calculate the environmental responsibility index for each company. Secondly, scholars may rely on environmental responsibility indices that other institutions have published. Considering the subjectivity of content analysis and data availability, this study selects the environmental responsibility index published by Hexun.com for the years 2010–2020 as the dependent variable. The main data processing and screening tools used in this paper are SPSS 23 and Stata 17.

#### Interpretive variables

The independent variable in this study is the implementation of a low-carbon economic policy. The low-carbon economic policy aims to promote sustainable development and reduce carbon emissions by adjusting the economic and industrial structures. As the explanatory variable, researchers can use the implementation of low-carbon economic policy to explore the impact of government or policy interventions on CER. By studying the implementation and effects of policies, we can understand the incentivizing role of policies on corporate behavior and environmental responsibility.

As for the explanatory variable, a quasi-natural experiment is constructed using the low-carbon economic policy implemented in 2016. The variable "Treat" represents the treatment group, with a dummy variable value of 1 if the company’s registered location falls within the scope of the low-carbon economic policy implementation, and 0 otherwise. The variable "Post" is a dummy variable for policy implementation, with a value of 1 for the years from 2016 onwards, and 0 otherwise.

#### Control variable

To address the issue of omitted variables, this study controls for other factors that may influence the level of CER as control variables. Following the study by Qin et al. (2018), the following indicators are selected as control variables in this study:

State Ownership (SOA): A dummy variable with a value of 1 if the company is state-owned and 0 otherwise. (1) Debt Ratio (Lev): Calculated as total liabilities divided by total assets. (2) Firm Size (Size): Measured by taking the logarithm of total assets. (3) Company Age (Age): Calculated as the current year minus the year of establishment. (4) Return on Assets (ROA): Calculated as net profit divided by the average total assets. (5) Board Size (Board size): Measured by the total number of board members. (6) Proportion of Independent Directors (Ind board): Calculated as the number of independent directors divided by the total number of board members. (7) Separation of Ownership and Control (Separation): The difference between the actual controlling shareholder’s control rights and ownership rights. (8) Concentration of Ownership (Top 1): The proportion of shares held by the largest shareholder.

### Design of the model

In this study, the implementation effect of low-carbon economic policy is evaluated based on the level of CER. Therefore, this study uses the Difference-in-Differences (DID) model as the main model. The model specification is explained below;

The variable “P(CERit = 1)”, otherwise termed CER-P, represents environmentally beneficial products and is treated as a dummy variable. It takes a value of 1 if a company applies or develops innovative products, technologies, or equipment that are beneficial to the environment, and 0 if otherwise. As the dependent variable is categorical or qualitative in nature, the model is based on a qualitative response regression model. The variable CERit measures the level of CER for firm i in year t. Treat is a dummy variable that separates the treatment group from the control group. If a firm implements the low-carbon economic policy, Treat takes a value of 1; otherwise, it takes a value of 0. Post is a dummy variable that distinguishes the post-treatment period from the control period. If the observation year is after 2016, Post takes a value of 1; otherwise, it takes a value of 0.

The coefficient α of Treat × Post reflects the relationship between the implementation of the low-carbon economic policy and the fulfillment of CER, which is the focus of this study. A positive coefficient would demonstrate that the implementation of the low-carbon economic policy promotes an increase in the level of CER. Conversely, a negative coefficient would indicate that the implementation of the low-carbon economic policy inhibits the fulfillment of CER. CV refers to the set of control variables in this study. Detailed explanations of each variable can be found in the previous text or in Table 1 variable definitions.

**Table 1:** Variable definitions.

Variable	Definitions
CER	Proxy variables for the level of corporate environmental responsibility. It takes a value of 1 if a company applies or develops innovative products, technologies, or equipment that are beneficial to the environment, and 0 otherwise.
Post	The experimental period and control period are divided. If the enterprise is in after 2016, the value is 1; otherwise, the value is 0
Treat	The experimental group and the control group are divided into two groups. If the region where the enterprise is registered is affected by low-carbon economic policies, the value is 1; otherwise, the value is 0
SOA	Whether it is state-owned or not, dummy variable, if it is a state-owned listed company, the value is 1, otherwise it is 0
Lev	The asset-liability ratio is calculated by dividing total liabilities by total assets.
Size	Company size, measured as logarithm of total assets
Age	The natural logarithm of company age
ROA	The net profit rate of total assets is calculated by dividing net profit by the average balance of total assets.
Ind board	The proportion of independent directors is calculated by dividing the number of independent directors by the total number of directors.
Separation	The degree of separation of two rights, the difference between control and ownership of the actual controller
Top1	Ownership concentration is the proportion of the largest shareholder.

## Results

### Descriptive statistics

This study provides a basic descriptive analysis of the main variables using a selected sample of companies, as shown in Table 2. The Table portrays that the mean value of CER is 0.435, with a standard deviation of 0.496. This data indicates the fact that most of the companies fail to meet the average level of environmental responsibility performance. There is a significant disparity in environmental responsibility performance among different companies, and overall, the level of environmental responsibility performance in the sample companies is not high. The mean value of Treat×Post is 0.184, with a standard deviation of 0.388. The median value is 0, which is below the average value of Treat×Post, indicating that more than half of the companies are not affected by the low-carbon economic policies. Among the control variables, the mean value of State-Owned Enterprises (SOE) is 0.511, indicating that half of the companies in the sample are state-owned enterprises. The characteristics of other variables are not significantly different from previous studies.

**Table 2:** Descriptive statistics.

Variable	Obs.	Mean	Std. dev.	median	Min	Max
CER	3,799	0.435	0.496	0.000	0.000	1.000
Post	3,799	0.572	0.495	1.000	0.000	1.000
Treat	3,799	0.320	0.466	0.000	0.000	1.000
Post*Treat	3,799	0.184	0.388	0.000	0.000	1.000
SOA	3,799	0.511	0.500	1.000	0.000	1.000
Lev	3,799	0.467	0.208	0.474	0.013	1.957
Size	3,799	22.542	1.393	22.323	18.370	26.918
Age	3,799	2.835	0.381	2.890	0.000	3.807
ROA	3,799	0.036	0.069	0.036	-1.395	0.482
Indboard	3,799	0.371	0.052	0.333	0.231	0.667
Separation	3,799	6.086	9.596	0.000	-69.493	50.000
Top1	3,799	37.519	16.440	35.78	0.000	90.000

### Correlation test

Table 3 presents the Spearman correlation coefficient matrix for the explanatory variables and major control variables. The absolute values of the correlation coefficients between variables do not exceed the empirical threshold of 0.7, indicating the absence of multi-collinearity issues among the variables. The absolute values of the correlation coefficients between the explanatory variables and control variables are all below 0.4, further indicating that the coefficient estimation of the explanatory variables will not be significantly affected by multi-collinear issues.

**Table 3:** Spearman correlation matrix.

Variables	CER	Post*Treat	SOA	Lev	Size	Age	ROA	Ind. board	Sep.	Top1
CER	1.000									
Post*Treat	0.161***	1.000								
SOA	0.192***	-0.008	1.000							
Lev	0.120***	0.016	0.391***	1.000						
Size	-0.002	0.154***	0.347***	0.518***	1.000					
Age	0.079***	0.212***	0.202***	0.133***	0.226***	1.000				
ROA	0.044***	0.012	0.204***	0.457***	0.039**	0.069***	1.000			
Indboard	0.018	0.033**	0.080***	0.042**	0.018	0.006	0.013	1.000		
Sep.	0.005	0.008	0.126***	0.035**	0.086***	0.051***	0.021	0.025	1.000	
Top1	0.101***	0.023	0.166***	0.096***	0.252***	0.064***	0.058***	0.058***	0.104***	1.000

Note:

*** p<0.01,

** p<0.05,

* p<0.1

### Parallel trend test

To ensure the non-biased estimation of results, the use of Difference-in-Differences (DID) regression requires the parallel trends assumption. In the context of this study, the parallel trends assumption refers to the dynamic impact of low-carbon economic policy on CER performance before and after the implementation of low-carbon economic policies [64]. The term "dynamic effect" describes how CER performance substantially enhances over time.

Fig 3 data shows that up until 2016, the environmental responsibility performance trends for both the experimental and control groups remained relatively steady. However, post-2016, the experimental group shows a distinct upward trend in CER performance. This indicates that only a limited number of companies demonstrated minimal CER efforts before the implementation of the low-carbon economic policy. Conversely, after the implementation, the policy compels companies to actively engage in CER activities, such as developing innovative products, technologies, or equipment that positively contribute to the environment.

**Fig 3:** Parallel trend test.

### Regression analysis

#### Low carbon economic policy and CER performance level

Table 4 shows the results of the baseline regression using fixed effects. The table explains that the variable PostTreat has a 0.100 coefficient at a significance p-value of 0.026***, indicating a significant effect at a certain level. This suggests that Post*Treat has a significant impact on CER. Again, researchers found the overall R2 of the experimental and control groups of the regression model to be 0.158. It demonstrates that the implementation of low-carbon economic policies can have a positive influence on the level of environmental responsibility performance by businesses. Implementing low-carbon economic policies is beneficial for enhancing the fulfillment of environmental responsibility by businesses, thus supporting Hypothesis 1.

**Table 4:** Baseline regression results.

	(1)	(2)	(3)	(4)	(5)	(6)	(7)	(8)	(9)
Post*Treat	0.312***	0.309***	0.310***	0.197***	0.104***	0.100***	0.100***	0.100***	0.100***
	(0.025)	(0.025)	(0.025)	(0.025)	(0.026)	(0.026)	(0.026)	(0.026)	(0.026)
Soa		0.135***	0.136***	-0.094**	-0.033	0.033	0.029	0.037	0.038
		(0.039)	(0.039)	(0.038)	(0.038)	(0.038)	(0.038)	(0.040)	(0.040)
Lev			0.029	0.176***	-0.073	-0.147**	-0.151**	-0.150**	-0.148**
			(0.063)	(0.063)	(0.061)	(0.071)	(0.071)	(0.071)	(0.071)
Size				0.200***	0.045**	0.052***	0.054***	0.054***	0.055***
				(0.014)	(0.018)	(0.018)	(0.018)	(0.018)	(0.018)
Age					0.581***	0.571***	0.566***	0.567***	0.563***
					(0.041)	(0.041)	(0.041)	(0.041)	(0.043)
Roa						-0.245**	-0.246**	-0.245**	-0.244**
						(0.120)	(0.120)	(0.120)	(0.120)
Indboard							0.282	0.274	0.272
							(0.176)	(0.177)	(0.177)
Seperation								-0.001	-0.001
								(0.001)	(0.001)
Top1									-0.000
									(0.001)
Constant	0.378***	0.447***	0.434***	3.982***	2.190***	2.288***	2.410***	2.409***	2.414***
	(0.008)	(0.022)	(0.035)	(0.318)	(0.333)	(0.336)	(0.345)	(0.345)	(0.345)
Obs	3,799	3,799	3,799	3,799	3,799	3,799	3,799	3,799	3,799
R-squared	0.046	0.049	0.049	0.103	0.156	0.157	0.158	0.158	0.158
No of id	525	525	525	525	525	525	525	525	525

**Note**: Standard errors in parentheses;

*** p<0.01,

** p<0.05,

* p<0.1

#### Mediation effect: Role of financing constraint

This study tested the mediation effects using the method proposed by [65], combined with the mediation effects testing method for Difference-in-Differences (DID) models by [66]. There are various ways in the academic community to measure financial constraints, mainly categorized into single-indicator or composite-indicator approaches. Single indicators include variables such as dividend payout ratio, interest coverage ratio, and firm size. Composite indicators include the KZ index, SA index, WW index, etc. In this study, the construction method of the Scale-Age Index (SA index) for measuring financial constraints, as developed by [67] was adopted. The SA index is the financial constraints of a firm that decrease the business growth in scale and has a longer operating period. It is widely recognized and used by many scholars in the field of financial constraint research and is considered representative. Therefore, this study used the SA index to measure the financial constraint variable.

Table 5 shows the regression models for examining mediation effects. The model shows that the R2 of the mediation variable SA index is 0.801, indicating that low-carbon economic policies positively impact financial constraints, which in turn affects the level of corporate environmental and social responsibility. The results validate Hypothesis 2, indicating that financial constraints mediate the relationship between low-carbon economic policies and the level of environmental responsibility.

**Table 5:** Coefficients of mediation regression model.

VARIABLES	(1)	(2)	(3)
	CER	SA index	CER
SA index			-0.365***
			(0.109)
Post*Treat	0.100***	-0.025***	0.091***
	(0.026)	(0.004)	(0.026)
Soa	-0.038	0.009	-0.034
	(0.040)	(0.006)	(0.040)
Lev	-0.148**	0.087***	-0.117
	(0.071)	(0.011)	(0.072)
Size	0.055***	-0.028***	0.045**
	(0.018)	(0.003)	(0.019)
Age	0.563***	-0.474***	0.390***
	(0.043)	(0.007)	(0.067)
Roa	-0.244**	0.047**	-0.227*
	(0.120)	(0.019)	(0.120)
Indboard	0.272	0.005	0.273
	(0.177)	(0.028)	(0.177)
Separation	-0.001	-0.001***	-0.001
	(0.001)	(0.000)	(0.001)
Top1	-0.000	-0.000	-0.000
	(0.001)	(0.000)	(0.001)
Constant	-2.414***	-1.860***	-3.094***
	(0.345)	(0.055)	(0.400)
Observations	3,799	3,799	3,799
R-squared	0.158	0.801	0.161

Note: Standard errors in parentheses;

*** p<0.01,

** p<0.05,

* p<0.1

### Probability of outcome and robustness test

This section of the research outlines the probability of the outcome for the dummy dependent variable and assesses the robustness using three widely recognized regression methods. Researchers employed the probit model to depict the probability outcome of a categorical variable, signifying the impact of low-carbon economic policy implementation on the expansion of CER activity in companies. Researchers applied a random effects model to accommodate panel data structures and address collinearity issues within the model. Researchers utilized Feasible Generalized Least Squares (FGLS) regression to attain more efficient and unbiased estimates, particularly when heteroscedasticity violations are present. The specific model is represented by the following formula.

Table 6 shows that the coefficient of the interaction term Treat×Post on environmentally beneficial products (CER-P) is significantly positive at 0.442. This suggests that the implementation of low-carbon economic policies contributes to an increased likelihood of companies developing or adopting innovative products, technologies, or equipment that are beneficial to the environment. In other words, the implementation of low-carbon economic policies facilitates the improvement of CER, consistent with the findings from the main regression analysis, thereby providing further validation of Hypothesis 1.

**Table 6:** Probability of outcome and robustness test.

VARIABLES	(1)	(2)	(3)
	Probit	RE	FGLS
Post*Treat	0.442***	0.148***	0.168***
	(0.056)	(0.023)	(0.021)
Soa	-0.516***	-0.178***	-0.193***
	(0.049)	(0.027)	(0.018)
Lev	-0.830***	-0.220***	-0.300***
	(0.142)	(0.061)	(0.052)
Size	0.112***	0.060***	0.041***
	(0.020)	(0.011)	(0.007)
Age	0.262***	0.359***	0.097***
	(0.059)	(0.029)	(0.022)
Roa	-0.798**	-0.292**	-0.292**
	(0.366)	(0.116)	(0.132)
Indboard	-0.039	0.237	-0.008
	(0.405)	(0.162)	(0.149)
Seperation	-0.003	-0.001	-0.001
	(0.002)	(0.001)	(0.001)
Top1	-0.006***	-0.001**	-0.002***
	(0.001)	(0.001)	(0.000)
Constant	-2.563***	-1.796***	-0.438***
	(0.433)	(0.224)	(0.157)
Observations	3,799	3,799	3,799

Note: Standard errors in parentheses;

*** p<0.01,

** p<0.05,

* p<0.1

Furthermore, the variable "Age" demonstrates a significant positive coefficient of 0.262 on environmentally beneficial products (CER). This indicates that older companies tend to be pioneers in implementing low-carbon economic policies, taking proactive steps to incorporate environmentally beneficial products in order to contribute to environmental protection. The random effect signifies the panel data structure, and researchers tested the model’s significant robustness using the FGLS, contributing more efficient and unbiased estimates for the control variables.

## Discussion

Global climate change and resultant sustainable practices have leveraged the intersection of low-carbon economic policies and corporate environmental responsibility (CER). The SDGs require that governments across the world devise and implement policies that help reduce carbon emissions. Such practices will bind corporations to strictly observe CER. However, firms deal with financial constraints that restrict their ability to implement such policies in true spirits. In this context, the study illuminates and presents its findings for understating and policy implementations. The study analyzes how the low-carbon economic policy has an impact on CER while keeping in view the financial accessibility and constraints of firms.

The study confirms that the introduction of low-carbon economic policies in 2016 has a positive effect on enhancing CER among Chinese A-share listed companies. Similar results that digital economic development depends on sustainable drives were found by Chen [55]. The implementation of low-carbon economic policies is positively correlated with the level of CER. Thus, it is understandable that the implementation of low-carbon economic policies can promote the level of CER in the pilot areas.

At the same time, the confirmation of Hypothesis 1 indicates the effectiveness of low-carbon economic policies in promoting corporate environmental governance, which is similar to the conclusions reached in the existing literature on the relationship between environmental regulations and corporate green governance [68, 69]. This indicates that firms are positively responding to governmental pressures or regulatory obligations that will ultimately reduce carbon emissions and promote sustainable business practices. Companies are incentivized to conform their operations with environmental standards by such regulations which encourage industry to adopt greener practices and promote sustainability [70]. Because firms are more likely to incorporate environmental responsibility into their strategic objectives by restructuring economic and industrial frameworks to prioritize emission reductions and resource efficiency [71]. In a market where sustainability is becoming more and more integral, this alignment not only helps businesses comply with regulations but also improves their reputation and competitiveness.

The validation of Hypothesis 2 underscores the importance of targeted policy interventions aimed at alleviating financial constraints faced by companies. The finding suggests that the impact of low-carbon policies on CER is conditioned by the firms’ financial capacity. Financial constraints as a bottleneck would make it difficult for companies to invest in green technology, comply with sustainable regulations and adopt sustainable practices. The impact of low-carbon economic policies on CER is a complex issue, and we find that financing constraints serve as an intermediary variable to explain this impact. Our finding is supported by [72] who stated that the implementation of low-carbon economic policies leads to a more favorable market perception of environment-friendly companies, as these companies can adapt to and comply with policy requirements and have a competitive advantage in future economic development. The companies may find it easier to obtain financing support, including bank loans and investments from investors. This financing support can help companies meet the requirements and investment needs of low-carbon economic policies. The result provides clear guidance to prioritize financial health as a part of firms’ environmental strategies.

The financing constraints are not the only intermediary variable, as other factors such as technological capabilities, management capabilities, and market demands may also play a mediating role in the impact of CER. Recognizing financial constraints as a mediator in the relationship between low-carbon policies and environmental responsibility underscores the importance of integrating financial support mechanisms into comprehensive sustainability strategies. This approach not only enhances regulatory compliance but also fosters a conducive environment for businesses to innovate and thrive in a sustainable future.

## Conclusion

This study discloses the complex dynamics between low-carbon economic policies, CER, and the role of financial constraints as a mediation. The relationships offer compelling evidence that though firms’ low-carbon policies are significant drivers of sustainable behavior, yet firm’s access to financial resources shapes their ability to fulfill environmental responsibilities. This study contributes to the understanding of how low-carbon economic policies influence Corporate Environmental Responsibility (CER) among Chinese A-share listed companies, specifically highlighting the role of financing constraints as a mediating factor. By employing a Difference-in-Differences (DID) model, the research confirms that the implementation of low-carbon economic policies since 2016 has positively impacted CER levels.

In conducting this research, careful consideration was given to alternative explanations, such as the influence of technological advancements and evolving market demands on Corporate Environmental Responsibility (CER). The study’s focus on financing constraints was chosen due to its relevance to the Chinese context, but other factors were acknowledged as significant and warrant further investigation. The researchers consciously reflected on their positionality, aiming to minimize any biases that could arise from their focus on economic and environmental policy intersections.

### Theoretical implications

The study’s contributions are multifarious. It strengthens the understanding of how low-carbon policies impact corporate behavior, while also providing a foundation for academic research exploring diverse mediators and broader contexts. Enriching corporate sustainability literature, the study elaborates climate-friendly policies, and corporate environmental performance amid the companies’ financial constraints. The study demonstrates that alleviating financial constraints enables companies to meet the heightened environmental standards set by these policies. The study highlights and adds to the stakeholders’ theory by showing how financial constraints facilitate meeting the environmental expectations of various stakeholders, including stockholders, governments, investors, and the general public.

Contributing to the institutional theory, the study acknowledges that firms’ responses to institutional pressures are not always the same but are constrained by financial factors. Organizations having limited resources may face these pressures, resulting in different levels of compliance. The results are in line with institutional theory which highlights the role of external regulatory and normative pressures in shaping organizational behavior. In view of institutional theory, organizations often conform to societal norms, values, and regulations to maintain legitimacy and social acceptance. Low-carbon policies are typically driven by government regulations, societal expectations, and market incentives which create a framework that incentivizes corporations to engage in environmentally responsible practices. This alignment reinforces the idea that corporate actions are influenced not just by economic goals, but also by the need to adhere to institutionalized environmental norms. However, this can also challenge institutional theory if the implementation of these policies results in superficial or symbolic compliance (institutional isomorphism) without substantive internal change, thereby questioning the depth of the institutionally-driven environmental commitment.

### Practical implications

Practically, the study endorses that governments and policymakers should arrange tailored financial support to help firms with limited financial capacity to overcome their needs and comply with environmental regulations. Subsidies, grants, tax incentives or low-interest loans can alternatively finance the financially constrained firms. The study highlights the need for financial planning as part of firms’ broader sustainability strategies. Firms’ reputation and legitimacy can be enhanced if regulators consider Environmental, Social, and Governance factors and incorporate such policies. By promoting policies that incentivize sustainable practices, governments can create an ecosystem where businesses are motivated to exceed mere compliance, leading to more robust environmental outcomes. Corporate decision-makers can leverage this relationship to align their strategic objectives with societal expectations, thereby enhancing their competitive advantage while contributing to broader sustainability goals. Furthermore, stakeholders, including investors and consumers, can utilize this information to hold corporations accountable for their environmental commitments, ensuring that companies not only adopt low-carbon policies but also integrate them into their core operations. Ultimately, this result emphasizes the interconnectedness of policy, corporate strategy, and stakeholder engagement in advancing environmental responsibility initiatives.

### Limitations and avenues for future research

Acknowledging several limitations, the study provides a few points for future research. The primary focus of this study was on financing constraints, other factors, including technological capabilities and market demands, can be investigated as potential mediators. The study explored how enhanced financial accessibility enables firms to invest in sustainable practices and contribute to a more robust environmental governance framework. Future research should focus on the long-term effects of low-carbon policies across different industries and regions, as well as their impact on unlisted firms, to develop a more comprehensive understanding of sustainable development. Future studies can find additional factors as to how governance strategies can support both economic growth and environmental preservation.

## Supporting information

S1 Data (XLSX)

## References

[1] ChenY-p, FuB-j, ZhaoY, WangK-b, ZhaoMM, MaJ-f, et al. Sustainable development in the Yellow River Basin: Issues and strategies. Journal of Cleaner Production. 2020;263:121223.

[2] ChenXH, TeeK, ElnahassM, AhmedR. Assessing the environmental impacts of renewable energy sources: A case study on air pollution and carbon emissions in China. Journal of environmental management. 2023;345:118525. doi: 10.1016/j.jenvman.2023.118525 37421726

[3] IEA. Tracking Clean Energy Progress 2023 2023. https://www.iea.org/reports/tracking-clean-energy-progress-2023.

[4] NASA. Airborne Nitrogen Dioxide Plummets Over China 2020. https://earthobservatory.nasa.gov/images/146362/airborne-nitrogen-dioxide-plummets-over-china.

[5] SunG, LiuY, LiB, GuoL. Road to sustainable development of China: The pursuit of coordinated development between carbon emissions and the green economy. Journal of Cleaner Production. 2024;434:139833.

[6] IRENA. Renewable Capacity Statistics 2020 2020. https://www.irena.org/publications/2020/Mar/Renewable-Capacity-Statistics-2020.

[7] TianH, QinJ, ChengC, JaveedSA, ChuT. Towards low-carbon sustainable development under Industry 4.0: The influence of industrial intelligence on China’s carbon mitigation. Sustainable Development. 2024;32(1):455–80.

[8] AFCA-SAC. Asian Financial Cooperation Association (AFCA) 2024. https://www.afca-asia.org/Portal.do?method=memberDetailView&returnChannelID=29&resourceID=3.

[9] LiuX, WenS. Should financial institutions in China bear environmental responsibility? Basic facts, theoretical models and empirical tests. Econ Res. 2019;54:38–54.

[10] MartinPR, MoserDV. Managers’ green investment disclosures and investors’ reaction. Journal of Accounting and Economics. 2016;61(1):239–54.

[11] WuS, ZhangH, WeiT. Corporate social responsibility disclosure, media reports, and enterprise innovation: evidence from Chinese listed companies. Sustainability. 2021;13(15):8466.

[12] QiS, LinS, CuiJ. Can environmental rights trading market induce green innovation?—Evidence based on green patent data of listed companies in China. Economic Research Journal. 2018;53(12):129–43.

[13] TrumppC, EndrikatJ, ZopfC, GuentherE. Definition, conceptualization, and measurement of corporate environmental performance: A critical examination of a multidimensional construct. Journal of Business Ethics. 2015;126:185–204.

[14] PengB, TuY, WeiG. Can environmental regulations promote corporate environmental responsibility? Evidence from the moderated mediating effect model and an empirical study in China. Sustainability. 2018;10(3):641.

[15] KrausS, RehmanSU, GarcíaFJS. Corporate social responsibility and environmental performance: The mediating role of environmental strategy and green innovation. Technological forecasting and social change. 2020;160:120262.

[16] KhanMK, TrinhHH, KhanIU, UllahS. Sustainable economic activities, climate change, and carbon risk: an international evidence. Environment, Development and Sustainability. 2022;24(7):9642–64. doi: 10.1007/s10668-021-01842-x 34602852 PMC8475409

[17] LiS, ZhengX, LiaoJ, NiuJ. Low-carbon city pilot policy and corporate environmental performance: Evidence from a quasi-natural experiment. International Review of Economics & Finance. 2024;89:1248–66.

[18] LinH. Cross-sector alliances for corporate social responsibility partner heterogeneity moderates environmental strategy outcomes. Journal of Business Ethics. 2012;110:219–29.

[19] KhanIU, HameedZ, KhanSU, KhanMA. Green banking practices, bank reputation, and environmental awareness: evidence from Islamic banks in a developing economy. Environment, Development and Sustainability. 2024;26(6):16073–93.10.1007/s10668-023-03288-9PMC1015982437363011

[20] VanhammeJ, LindgreenA, ReastJ, Van PoperingN. To do well by doing good: Improving corporate image through cause-related marketing. Journal of business ethics. 2012;109:259–74.

[21] ChanTY, WongCW, LaiKH, LunVY, NgCT, NgaiEW. Green service: construct development and measurement validation. Production and Operations Management. 2016;25(3):432–57.

[22] CaiL, HeC. Corporate environmental responsibility and equity prices. Journal of Business Ethics. 2014;125:617–35.

[23] TettehLA, Agyenim-BoatengC, SimpsonSNY. Institutional pressures and accountability processes in pursuit of sustainable development goals: Insights from Ghanaian indigenous oil companies. Corporate Social Responsibility and Environmental Management. 2024;31(1):89–107.

[24] HuangY-C, HuangC-H. Exploring institutional pressure, the top management team’s response, green innovation adoption, and firm performance: evidence from Taiwan’s electrical and electronics industry. European Journal of Innovation Management. 2024;27(3):800–24.

[25] WanG, ZhangW, LiC. How does low-carbon city pilot policy catalyze companies toward ESG practices? Evidence from China. Economic Analysis and Policy. 2024;81:1593–607.

[26] Al-OmoushKS. Drivers of digital corporate social responsibility during unprecedented crises: an institutional perspective. Kybernetes. 2024;53(3):882–900.

[27] DiMaggio PJ. Interest and agency in institutional theory. Institutional Patterns and Organizations: Culture and Environment/Ballinger. 1988.

[28] NorthDC. The new institutional economics. Journal of Institutional and Theoretical Economics (jite)/Zeitschrift für die gesamte Staatswissenschaft. 1986;142(1):230–7.

[29] WangS, LiJ, RazzaqA. Do environmental governance, technology innovation and institutions lead to lower resource footprints: An imperative trajectory for sustainability. Resources Policy. 2023;80:103142.

[30] MaoX, WangY, ZameerH, SongH. Can Chinese outward foreign direct investment help the belt and road low-carbon development? Evolutionary game in China’s environmental responsibility. Environment, Development and Sustainability. 2024;26(5):11049–88.

[31] YaoH, WanZ, ZengH, WuQ. How Does Low-Carbon Financial Policy Affect Corporate Green Innovation?—Re-Examination of Institutional Characteristics, Influence Mechanisms, and Local Government Behavior. Sustainability. 2024;16(10):3944.

[32] KhanSU, WangM, KhanIU, LiuXd. Evaluating stock trading behaviour: Information sources nexus through intrinsic and extrinsic motivation. International Journal of Finance & Economics. 2022;27(3):2965–76.

[33] WuR, LinB. Environmental regulation and its influence on energy-environmental performance: evidence on the Porter Hypothesis from China’s iron and steel industry. Resources, Conservation and Recycling. 2022;176:105954.

[34] PorterME, LindeCvd. Toward a new conception of the environment-competitiveness relationship. Journal of economic perspectives. 1995;9(4):97–118.

[35] SunX, ZhangR, YuZ, ZhuS, QieX, WuJ, et al. Revisiting the porter hypothesis within the economy-environment-health framework: Empirical analysis from a multidimensional perspective. Journal of Environmental Management. 2024;349:119557. doi: 10.1016/j.jenvman.2023.119557 37956516

[36] Brand-CorreaL, BrookA, BüchsM, MeierP, NaikY, O’NeillDW. Economics for people and planet—moving beyond the neoclassical paradigm. The Lancet Planetary Health. 2022;6(4):e371–e9. doi: 10.1016/S2542-5196(22)00063-8 35397225 PMC9226380

[37] MengB, ZangQ, LiG. Study on the impact of corporate social responsibility on carbon performance in the background of carbon peaking and carbon neutrality. Business Ethics, the Environment & Responsibility. 2024;33(3):416–30.

[38] LiH, BhattiZ, AbbasQ, AhmadI, IqbalN, AzizB. Measuring low carbon energy, economic and environmental sustainability performance of BRICS. The Singapore Economic Review. 2024;69(01):357–76.

[39] FoxonTJ. A coevolutionary framework for analysing a transition to a sustainable low carbon economy. Ecological economics. 2011;70(12):2258–67.

[40] ZhangZ. Making the transition to a low-carbon economy: the key challenges for China. Asia & the Pacific Policy Studies. 2016;3(2):187–202.

[41] SovacoolBK, NewellP, CarleyS, FanzoJ. Equity, technological innovation and sustainable behaviour in a low-carbon future. Nature human behaviour. 2022;6(3):326–37. doi: 10.1038/s41562-021-01257-8 35102347

[42] ChenY, RenY-S, NarayanS, HuynhNQA. Does climate risk impact firms’ ESG performance? Evidence from China. Economic Analysis and Policy. 2024;81:683–95.

[43] KlassenRD, WhybarkDC. Environmental management in operations: the selection of environmental technologies. Decision sciences. 1999;30(3):601–31.

[44] PanY, ChenQ, ZhangP. Does policy uncertainty affect corporate environmental information disclosure: evidence from China. Sustainability Accounting, Management and Policy Journal. 2020;11(5):903–31.

[45] SolikhahB, MaulinaU. Factors influencing environment disclosure quality and the moderating role of corporate governance. Cogent Business & Management. 2021;8(1):1876543.

[46] YiL, BaiN, YangL, LiZ, WangF. Evaluation on the effectiveness of China’s pilot carbon market policy. Journal of Cleaner Production. 2020;246:119039.

[47] KhanM, MajidA, YasirM, ArshadM. Corporate social responsibility and corporate reputation: A case of cement industry in Pakistan. Interdisciplinary Journal of Contemporary Research in Business. 2013;5(1):843–57.

[48] Luoma-ahoV. Corporate reputation and the theory of social capital. The handbook of communication and corporate reputation. 2013:279–90.

[49] LiF, GuoY, LiuB. Impact of government subsidies and carbon inclusion mechanism on carbon emission reduction and consumption willingness in low-carbon supply chain. Journal of Cleaner Production. 2024;449:141783.

[50] YeeW-H, TangS-Y, LoCW-H. Regulatory compliance when the rule of law is weak: Evidence from China’s environmental reform. Journal of Public Administration Research and Theory. 2016;26(1):95–112.

[51] BednarMK. Watchdog or lapdog? A behavioral view of the media as a corporate governance mechanism. Academy of Management Journal. 2012;55(1):131–50.

[52] WangF, SunZ, FengH. Can media attention promote green innovation of Chinese enterprises? Regulatory effect of environmental regulation and green finance. Sustainability. 2022;14(17):11091.

[53] RenS, ZhengJ, LiuD, ChenX. Does emissions trading system improve firm’s total factor productivity—Evidence from Chinese listed companies. China Ind Econ. 2019;5(05):5–23.

[54] CuiJ, DaiJ, WangZ, ZhaoX. Does environmental regulation induce green innovation? A panel study of Chinese listed firms. Technological Forecasting and Social Change. 2022;176:121492.

[55] ChenP. Corporate social responsibility, financing constraints, and corporate carbon intensity: new evidence from listed Chinese companies. Environmental Science and Pollution Research. 2023;30(14):40107–15. doi: 10.1007/s11356-023-25176-5 36609966 PMC9822695

[56] NaseemMA, LinJ, RehmanRU, AhmadMI, AliR. Moderating role of financial ratios in corporate social responsibility disclosure and firm value. PloS one. 2019;14(4):e0215430. doi: 10.1371/journal.pone.0215430 30998740 PMC6472779

[57] TianP, LinB. Impact of financing constraints on firm’s environmental performance: Evidence from China with survey data. Journal of Cleaner Production. 2019;217:432–9.

[58] AkbarA, JiangX, QureshiMA, AkbarM. Does corporate environmental investment impede financial performance of Chinese enterprises? The moderating role of financial constraints. Environmental Science and Pollution Research. 2021;28(41):58007–17. doi: 10.1007/s11356-021-14736-2 34101121

[59] WuC, WuS, ChengJ, WangL. The role of venture capital in the investment and financing behavior of listed companies: evidence from China. Economic Research Journal. 2012;47(1):105–19.

[60] JiangY. The cost of equity, the cost of debt and the corporate governance: a study on the difference in influence. J Manag World. 2009;11:144–55.

[61] HanS, PanY, MygrantM, LiM. Differentiated environmental regulations and corporate environmental responsibility: the moderating role of institutional environment. Journal of Cleaner Production. 2021;313:127870.

[62] TsalisTA, NikolaouIE, KonstantakopoulouF, ZhangY, EvangelinosKI. Evaluating the corporate environmental profile by analyzing corporate social responsibility reports. Economic Analysis and Policy. 2020;66:63–75.

[63] WangH. Corporate Social Responsibility in China. The Palgrave Handbook of Corporate Social Responsibility. 2020:1–24.

[64] WangJ ZY, CookeFL. Low-carbon economy and policy implications: a systematic review and bibliometric analysis. Environmental Science and Pollution Research. 2022;29(43): 65432–51. doi: 10.1007/s11356-022-20381-0 35486269

[65] WenZ, YeB. Analyses of mediating effects: the development of methods and models. Advances in psychological Science. 2014;22(5):731.

[66] ShiD, DingH, WeiP, LiuJ. Can smart city construction reduce environmental pollution. China Ind Econ. 2018;6:117–35.

[67] HadlockCJ, PierceJR. New evidence on measuring financial constraints: Moving beyond the KZ index. The review of financial studies. 2010;23(5):1909–40.

[68] AmoreMD, BennedsenM. Corporate governance and green innovation. Journal of Environmental Economics and Management. 2016;75:54–72.

[69] HuangL, LeiZ. How environmental regulation affect corporate green investment: evidence from China. Journal of Cleaner Production. 2021;279:123560.

[70] UllahS, KhanFU, AhmadN. Promoting sustainability through green innovation adoption: a case of manufacturing industry. Environmental Science and Pollution Research. 2022;29(14):21119–39. doi: 10.1007/s11356-021-17322-8 34746984

[71] UllahS, KhanFU, SaeedI. Promoting green growth through identification of sustainable strategies: a hybrid approach. International Journal of Emerging Markets. 2024.

[72] ZhangD, LuceyBM. Sustainable behaviors and firm performance: The role of financial constraints’ alleviation. Economic Analysis and Policy. 2022;74:220–33.

